This article has been retracted.

# Mesenteric Panniculitis: A Rare Condition in a Patient With Rheumatoid Arthritis

**DOI:** 10.7759/cureus.20136

**Published:** 2021-12-03

**Authors:** Thamer S Alzahrani, Ali H Alharbi, Abdulellah I Al Homoudi, Arwa A Reidi, Farah A Alshehri, Nawaf F Alsarraj, Heba H Milibary, Rashed A Alnemer, Yousef Z Murad, Sarah M Almousa, Bashaier M Albalawi, Ayman J Almalky, Ali B Alaithan, Furqan H Alawami, Faisal Al-Hawaj

**Affiliations:** 1 College of Medicine, Al-Baha University, Al-Baha, SAU; 2 General Practice, Al-Nakheel Primary Health Care Center, Qassim, SAU; 3 College of Medicine, Dar Al Uloom University, Riyadh, SAU; 4 College of Medicine, Ibn Sina National College for Medical Studies, Jeddah, SAU; 5 College of Medicine, King Abdulaziz University, Jeddah, SAU; 6 College of Medicine, King Saud Bin Abdulaziz University for Health Sciences, Riyadh, SAU; 7 College of Medicine, Tabuk University, Tabuk, SAU; 8 College of Medicine, Taif University, Taif, SAU; 9 College of Medicine, Vision Colleges, Riyadh, SAU; 10 College of Medicine, Imam Abdulrahman Bin Faisal University, Dammam, SAU

**Keywords:** case report, abdominal pain, computed tomography, mesenteric panniculitis, rheumatoid arthritis

## Abstract

Rheumatoid arthritis is a relatively common chronic inflammatory disorder affecting the synovial joints. Extra-articular manifestations of rheumatoid arthritis are not uncommon and include a wide range of cardiovascular, pulmonary, and neurological complications. Gastrointestinal involvement in rheumatoid arthritis is rare, but it can be impactful on the quality of life of patients. We present the case of a 45-year-old woman, with rheumatoid arthritis on methotrexate, who presented with a one-week history of abdominal pain. The patient visited the outpatient clinic earlier and was diagnosed with indigestion and was offered symptomatic treatment which failed to provide any improvement. Abdominal examination revealed a distended abdomen with generalized tenderness and rebound. However, the abdomen was soft with no palpable masses. Initial laboratory examination, including inflammatory parameters, was normal. The patient underwent a computed tomography scan of the abdomen with intravenous contrast which demonstrated inhomogeneous hyperdense mesenteric fat giving a mass-like lesion with a displacement of adjacent bowel loops. Such findings conferred the diagnosis of mesenteric panniculitis. The patient was started on corticosteroid therapy with oral prednisolone 40 mg daily with close follow-up. She developed gradual improvement in her condition and the pain resolved completely after six days. The patient was re-evaluated after six months from discharge and she had no recurrence. The case highlighted a rare association of mesenteric panniculitis and rheumatoid arthritis. Physicians should keep this mesenteric panniculitis in mind when they encounter patients with the autoimmune disorders who presented with abdominal symptoms.

## Introduction

Rheumatoid arthritis is a chronic polyarticular inflammatory disorder of unknown etiology that tends to affect small joints. The prevalence of rheumatoid arthritis reaches up to 1% of the population [1]. It is twice more common in women compared with men. While rheumatoid arthritis is primarily a disorder of synovial joints, extra-articular involvement may occur [1]. The risk factor for systemic involvement in rheumatoid arthritis include advanced age, smoking, positive rheumatoid factor or antinuclear antibody, and having human leukocyte antigen DRB1 alleles [2]. Extra-articular manifestations of rheumatoid arthritis, include renal, cardiovascular, pulmonary, and neurological manifestations [3]. However, gastrointestinal involvement in rheumatoid arthritis is rare, but it can be impactful on the quality of life of patients. It is reported that patients with rheumatoid arthritis exhibit a higher risk for having abnormal esophageal motility and reflux disease, chronic gastritis, and secondary amyloidosis [2]. Here, we present the case of a middle-aged woman with rheumatoid arthritis who developed mesenteric panniculitis, which is a rare association with few reported cases in the medical literature [3].

## Case presentation

We present the case of a 45-year-old woman who presented to the emergency department with a one-week history of abdominal pain. Her pain was located in the epigastric area and was non-radiating. She described the pain as constant and stabbing in nature. She scored it 7 out of 10 on the severity scale. The pain was not related to meals or posture. It was partially relieved by the over-the-counter analgesics. The pain was associated with nausea and vomiting. There was no history of change in bowel habits. The patient reported no history of anorexia or weight loss. She visited the outpatient clinic earlier for this pain and was diagnosed with indigestion and was offered symptomatic treatment which failed to provide any improvement.

The patient had a significant past medical history of rheumatoid arthritis. She was diagnosed at age of 34 years. The patient was using methotrexate for her disease for the last five years. She used naproxen 500 mg almost daily for her hand pain of arthritis. She also had a history of scalp psoriasis that was well-controlled with salicylic acid shampoo. The surgical history was remarkable for tonsillectomy only. The patient was a non-smoker and never consumed alcohol. She worked as an artist but had to quit her job because she lost her hand dexterity due to rheumatoid arthritis. Her family history was remarkable for autoimmune diseases.

Upon examination, the patient appeared tired and in discomfort. Her vital signs were within the normal limits, including a temperature of 37.5℃, pulse rate of 88 bpm, respiratory rate of 18 bpm, and blood pressure of 112/78 mmHg. Her oxygen saturation was normal. Abdominal examination revealed a distended abdomen with generalized tenderness and rebound. However, the abdomen was soft with no palpable masses. Abdominal auscultation revealed normal bowel sounds with normal intensity and frequency. Examination of other systems was non-contributory.

Initial laboratory examination included hemoglobin level of 14.2 g/dL, white cell counts of 8500/μL, and platelets count of 380,000/μL. She had normal levels of erythrocyte sedimentation rate and C-reactive protein. The liver and kidneys profiles were within the normal limits (Table 1). While the laboratory markers were reassuring, the treating physician was concerned about the physical examination findings and suggested further investigation with imaging studies.

**Table 1:** Summary of the results of laboratory findings

Laboratory Investigation	Unit	Result	Reference Range
Hemoglobin	g/dL	14.2	13.0–18.0
Leukocytes	1000/mL	8.5	4.0–11.0
Platelet	1000/mL	380	140–450
Erythrocyte Sedimentation Rate	mm/hr.	14	0–20
C-Reactive Protein	mg/dL	7.1	0.3–10.0
Total Bilirubin	mg/dL	0.4	0.2–1.2
Albumin	g/dL	3.9	3.4–5.0
Alkaline Phosphatase	U/L	58	46–116
Gamma-glutamyltransferase	U/L	24	15–85
Alanine Transferase	U/L	19	14–63
Aspartate Transferase	U/L	20	15–37
Blood Urea Nitrogen	mg/dL	11	7–18
Creatinine	mg/dL	0.8	0.7–1.3
Sodium	mEq/L	138	136–145
Potassium	mEq/L	3.9	3.5–5.1
Chloride	mEq/L	104	98–107

The patient underwent a computed tomography scan of the abdomen with intravenous contrast. The scan demonstrated inhomogeneous hyperdense mesenteric fat giving a mass-like lesion with a displacement of adjacent bowel loops. It was notable that the fat surrounding the mesenteric vessels was spared giving the appearance of a fat ring sign. Multiple enlarged mesenteric and retroperitoneal lymph nodes. Such findings conferred the diagnosis of mesenteric panniculitis (Figures 1, 2).

**Figure 1:** Axial CT image demonstrates inhomogeneous lesion of adipose tissue (arrows) sparing the adjacent mesenteric vessels. CT: computed tomography

**Figure 2:** Coronal CT image demonstrates inhomogeneous hyperdense mesenteric fat sparing the mesenteric vessels giving the appearance of fat ring sign. CT: computed tomography

The patient was started on corticosteroid therapy with oral prednisolone 40 mg daily with close follow-up. She developed gradual improvement in her condition and the pain resolved completely after six days. She was discharged after 10 days of hospitalization. The patient had regular follow-up visits for her condition. The corticosteroid therapy was continued for two months. The patient was re-evaluated after six months from discharge and she had no recurrence or new complaints.

## Discussion

We reported a rare case of mesenteric panniculitis in a middle-aged woman with rheumatoid arthritis. Mesenteric panniculitis is a rare idiopathic inflammatory condition affecting the adipose tissue [4]. It typically involves the small intestine mesentery, but the large intestine can be involved on rare occasions. The true prevalence of this condition is unknown, but a prior study indicated that it is less than 1% [5].

While the pathogenesis of mesenteric panniculitis is unclear, certain clinical factors have been shown to have a significant association with this condition. Such diseases included autoimmune disorders, infections, malignancies, and hypersensitivity reactions. In the present case, mesenteric panniculitis occurred in the setting of rheumatoid arthritis [5]. We assume that the development of mesenteric panniculitis in our patient could be related to her underlying disease directly or because of its treatment [6]. A previous study indicated that methotrexate was associated with panniculitis [7].

In contrast to the present case, mesenteric panniculitis is often asymptomatic and is detected incidentally on cross-sectional studies performed for other indications [4]. However, patients may present with a broad spectrum of manifestations, including abdominal pain and a palpable mass. The laboratory investigations, including the inflammatory parameters, lack the sensitivity and specificity to make the diagnosis of panniculitis [6]. There are many conditions that may present with a similar clinical picture to that of mesenteric panniculitis. Such conditions include a wide range of malignancies [5]. Hence, a computed tomography scan is of paramount importance to diagnose this disorder. As our patient’s scan has demonstrated, the mesenteric panniculitis manifests radiologically as inhomogeneous adipose tissue that does not invade the surrounding bowel loops and spared the mesenteric vessels.

Regarding the management of this disorder, no indication is advised if the patient is asymptomatic as the disease resolves spontaneously. However, in the present case, the patient was given corticosteroid therapy and had a successful response. Surgical management can be attempted if the patient failed to respond to medical treatment [6].

## Conclusions

The case highlighted a rare association of mesenteric panniculitis and rheumatoid arthritis. Physicians should keep this mesenteric panniculitis in mind when they encounter patients with autoimmune disorders who presented with abdominal symptoms. Cross-sectional imaging studies are crucial in making the diagnosis because of its non-specific features. Medical treatment with corticosteroid therapy is usually successful for the management of this condition.
